RETRACTED

# On the Professional Development Environment of Young Teachers in the Series of Quality Education in Colleges and Universities

**DOI:** 10.1155/2022/5370757

**Published:** 2022-08-22

**Authors:** Zhengnan Qi

**Affiliations:** Zhejiang Agricultural Business College, Shaoxing 321088, China

## Abstract

With the changes of the times, China has made remarkable achievements in economic, political, social, cultural, and education can improve the comprehensive quality of the people, enhancing the country's comprehensive national strength and international competitiveness effect. China has importance to education, and in recent years has increased its investment in education. Higher education undertakes important functions such as cultivating talents, scientific research, and serving the society. It is an indispensable part of the education system, and these are closely related to the teaching staff of colleges. The development of quality education is an inevitable choice to promote it, an important way to implement it with morality, and promoting it of national governance capabilities. At present, there are four major problems in quality education in colleges: the marginalization of status, fuzzy goals, segmentation of content, and isolation of development paths. It is important to study and explore new ideas and strategies for promoting quality education. Nowadays, colleges are no longer the “ivory towers” of the past, and the construction of college teachers has also undergone many changes compared with the past. The topics and discussions about college teachers are increasing day by day, and the problems and confusion exposed to them have also aroused the attention of the society. Young teachers are the fresh blood of college teachers and the future of our country. It is particularly meaningful to study and understand the current professional development of these groups. The research object is the young teachers in colleges. Through the literature research method, it analyzes the status of the professional quality education in colleges, understands the problems existing in their professional development, analyzes the reasons, and puts forward corresponding countermeasures. It helps for the career development of the whole group of young teachers in colleges in order to improve the current situation, seek better development for young teachers in colleges, and also provide a reference for promoting quality education in colleges.

## 1. Introduction

At present, China's higher education is gradually transforming from its basic supporting role of it to supporting and leading the development [1]. Only by actively studying and discussing the direction and new strategies of implementing quality education can colleges and universities truly implement them, provide a solid foundation for cultivating excellent and top-notch talents, and truly shoulder the responsibilities and tasks of education [2]. It provides intellectual and talent support [3].

RETRACTED

As China develops into a large socialist democratic country led by the Communist Party of China in the world, it also determines that our higher education system should take the training of great social party builders and successors as its basic tasks, try its best to train a number of useful Chinese people from generation to generation, support the leadership of the Communist Party and China's socialist democratic system, and they will be determined to work hard for China's socialist development forever. He pointed out the direction for the innovative development of quality education for college students [4]. It can promote the prosperity and development of various undertakings of the central leading collective, and follow up talents. It is also conducive to promoting lofty education and realizing the lofty ideal of socialismhow to grasp the fundamental of education completely and correctly [5]. Actively promote quality education, bring up excellent graduates who meet the needs of the new era, correct some deviations in the theory and implementation of quality education,and promote the harmonious unity of vocational education and quality education. It is the central topic of school education research [6].

As a unique quasi public service industry, higher education can provide huge public services to the public, and the participants in the field of higher education have a great impact on it [7]. The number of young teachers participating in higher education continues to expand. The main work of these professors is to train professional knowledge, cultivate excellent talents and participate in research projects.  Figure 1 shows the development and world level of young teachers in China from 2009 to 107 [8]. Noble and selfless the teacher profession in the past thought, in the modern society, teachers have become a unique rational education subject after entering the education cause. Therefore, their actual professional play will play an important role in the performance of the teaching cause [9]. Low professional title and insufficient experience. Therefore, in this study, the key is to analyze in detail the professional work of young college teachers after they participate in social work [10].

The quality of education in colleges is largely limited by the level of efficient teachers [11]. Before, the number of young teachers in Chinese colleges and universities increased significantly[12]. Young teachers have gradually evolved into the main force of higher education in the new era, and they are also the most important force. It is extremely important to recognize the current professional development status and problems of young teachers. The essential. In practical activities, the stability of college teachers' teams and the development of the education system are closely related to young teachers. The career development of young teachers has a significant impact on their actual performance in teaching and research. However, for the young teachers in the current university, some of them are relatively old, have relatively shallow education experience, and have strict promotion requirements. They cannot emphasize the importance of education, and the actual pressure is relatively large [13].

RETRACTED

## 2. Theoretical Research

### 2.1. The Connotation and Significance of Quality Education in Colleges

#### 2.1.1. The Connotation of Quality Education in Colleges

Quality education refers to a policy that aims at improving personal quality, focuses on cultivating students' basic spirit and practical quality, and includes science, morality, art, and discipline as the basis to create students' morality, intelligence, physique, and discipline [14]. From the perspective of pedagogy, education lays more emphasis on basic functions, which refers to the sum of those stable, basic, social evaluation, and other meaningful characteristics, which can have a wide impact on the efficiency of human life and the future development of society [15].

Before the reform and opening up, education had been interfered by the “left” education trend at that time. The students were not good enough and could not serve politics; after the reform and opening-up, the school has received the impact of examination oriented education. The most important thing is the curriculum, but it has neglected the cultivation and promotion of humanistic ethics [16]. The proposal of quality education clarifies the ontological function of quality education, that is to improve the quality of education itself [17]. It is necessary to take positive measures to promote the organic integration of human creativity, practical skills, and entrepreneurial spirit, so as to improve the overall improvement of human cultural literacy and scientific and technological ability [18]. In July 2010, the “National Medium- and Long-Term Education Reform and Development Plan (2010–2020)” issued by the Ministry of Education once again identified the popularization of high-quality higher education as a national key topic. Since then, the central government has made a series of resolutions on strengthening and improving the quality of higher education. He pointed out: “We must fully implement the Party's educational policy, implement the fundamental task of morality and cultivating people, and develop quality Education, promote education fairness, and cultivate socialist builders and successors with all-round development of morality, intelligence, physique, and beauty.” The 2018 National Undergraduate Education Work Conference pointed out that undergraduates in colleges should be the principle of “based on this” and promote the “four a return”. This has an important and far-reaching impact on it higher education, especially the training of talents. The meeting emphasized that students should be guided to read traditional cultural classics and read “national books”, which provided strong policy support for promoting quality education.  Figure 2 is China's 2017 -Market situation in the quality education industry in 2023 [19].

RETRACTED

#### 2.1.2. The Significance of Quality Education in Colleges

Developing aesthetic education is a necessary option to further improve the quality of primary and middle school students [20]. Higher education has the dual role of promoting its own growth and comprehensive development. Improving its own growth is the basis for higher education and promoting social progress [21]. The basic purpose of school education is to cultivate student information technology knowledge and innovation ability, good personality quality, positive psychological quality to cope with social changes, and innovative quality to be competent for the post. This also shows that the essence of the development of university education is to improve the quality education of Chinese college students and stimulate the power and vitality of the sustainable development of college students.

Developing quality education is an important way. Developing quality education is the requirement of the times for policy. Through the concept of educational socialism, adhere to the combination of “moral education first and people-oriented”, carry forward the Chinese spirit, enhance “four kinds of self-confidence,” cultivate patriotism, civic will and lofty ideological and moral quality, and improve the “entrepreneurial spirit, ability and socialist sense of responsibility” of College students by using diversified education strategies. Quality education focuses on improving the comprehensive quality of their quality, cultural and scientific quality, professional skills quality, and so on to establish values so that they can become students with both political integrity and comprehensive development talents, to promote it.

### 2.2. The Connotation of the Career Development of Young Teachers in Colleges

#### 2.2.1. Young Teachers in Colleges

Young teachers in Institutions of higher learning refer to full-time public institutions of higher learning that provide academic education or training for junior college, undergraduate or higher education, including comprehensive institutions of higher learning, vocational colleges and other ordinary colleges and universities, excluding specialized personnel in adult higher education. As for the specific judgment of young teachers, age is one of the key factors, but there is currently no unified standard worldwide: the United Nations considers the age of young people to be between 15–24 years old; UNESCO defines it as 16–24 years old. 45 years of age; the revised WHO definition is 18–65 years old; and the Chinese Bureau of Statistics standard is 15–34 years old. Concerning the current structural system of college teachers and various materials issued by it, the age stage of young teachers in colleges is finally determined to be less than 40 years old. Because the definition of college teachers is more complex, in the analysis of the paper, the focus is on the front-line full-time teachers who participate in teaching and research work.

RETRACTED

#### 2.2.2. Career Development Theory

Career theory plays an important role in guiding each person's career development in life. Many scholars around the world have carried out analyses based on multiple perspectives and then formed their career theories. Overall, there are mainly career choice and development theories.

The core of the theory of choice is the “career person matching theory” proposed by Parsons. The core of this concept is that, on the one hand, people must understand their own interests, preferences and needs, and at the same time, they must understand the specific characteristics and conditions of things.

These ideas are all studied from the individual point of view. Foreign scholars focus on age, so their career can be divided into different stages. And so on, gave their own career development concept. After studying various concepts, we conclude that the concept of Shi en has a relatively detailed definition of the individual's growth stage, and there is time overlap, as shown in Table 1.

The analysis of Chinese scholar Liao Quanwen is different from the age-based development theory of overseas scholars, and a new “three three three” theory has been formed, as shown in Table 2 below.

## 3. Research on the Current Situation of Quality Education in Colleges and the Professional Development of Young Teachers

### 3.1. The Current Development Dilemma of Quality Education in Colleges

#### 3.1.1. The Status of Quality Education is Marginalized

It believes that “emphasizing people-oriented teaching and promoting overall aesthetic education is a strategic issue for the growth of the school.” From the perspective of our country's policy, the important strategic position of aesthetic education as a national strategic theme has been determined, and actively promoting aesthetic education has become the important significance and inevitable condition for the priority development of socialist higher education. However, the practice has proved that although the current aesthetic education in Chinese colleges and universities has made certain achievements, there are still defects and imbalances in the development status, there are huge differences between the development quality and social needs, and the important strategic position of aesthetic education and the scientific research evaluation system have not been properly set up.  Figure 3 shows China's current development level of students' quality education in colleges at all levels.

RETRACTED

#### 3.1.2. The Effective Integration of Quality Education and Higher Education has not been Achieved

It also has many fine traditions, such as paying attention to the optimization of the curriculum and the strict teacher training system. However, due to the influence of examination oriented education, some teachers often only bear the cost of professional knowledge and rarely apply the teaching content to the implementation of quality education, thus causing students to have a superficial and incomplete understanding of the education content and doing nothing to improve their own moral quality. The impact of quality education is very extensive. Therefore, when we talk about the effective integration of quality education and higher education, we often talk about it verbally but do not implement it.

### 3.2. Current Situation of Career Development of Young Teachers in Colleges-Taking H University as an Example

#### 3.2.1. Basic Situation of Young Teachers in H University

Among the full-time teachers of H University, there are 247 young teachers aged 40 and below, accounting for 67.12% of the total number of it, including 17 deputy senior teachers, 123 intermediate teachers, 107 junior and undetermined teachers. (Table 3).

#### 3.2.2. Current Situation of Career Development of Young Teachers at H University

The research on the career development of their at H University involves all aspects of teachers' work, life, and learning. In this research, the author mainly conducts an in-depth study on this issue by investigating teachers' experiences and feelings on teaching, professional title evaluation, remuneration, training and other aspects.

RETRACTED

The statistical results in Table 4 show that the respondents' overall feeling about the profession of college teachers is the busiest choice (64.1%), followed by a sense of pride (49.5%), followed by very stressful (45.6%), and a sense of accomplishment (45.6%). It shows that the respondents feel that they are busy and stressed about the profession of college teachers, but they also affirm the sense of pride and achievement brought by this profession, which can also reflect a certain extent their commitment to the profession of college teachers. Overall evaluation: Hard work but good social prestige.

In Table 5, the statistical results of the factors affecting their career development selected by the respondents in order of importance are: scientific research level, academic resources, teaching level, interpersonal communication, work environment, and others. This also shows that the surveyed young teachers in colleges attach more importance to scientific research work, and the degree of emphasis is greater than that of teaching staff.

It can be seen from the above survey that teaching and scientific research are the two main aspects of college teachers' work. Combined with questionnaires, interviews, and the author's experience in actual work, it is a long-standing fact that most college teachers emphasize scientific research in their daily work.  Figure 4 shows the number of NS papers published by young teachers in colleges from 2003 to 2017. Scientific research activities are one of the main tasks of college teachers. Understandably young college teachers attach importance to scientific research. However, from the actual implementation and the different requirements for teaching and scientific research for professional title review itself, it can be found that teaching work is often used as workload statistics. Most schools and teachers pay more attention to scientific research work, and teachers often choose teaching work as a “task” is completed, and more time and energy are invested in scientific research. A person's energy is limited. After a lot of investment in scientific research activities, less is allocated to other work content, which affects the development of other work to a certain extent.

## 4. Countermeasures and Suggestions for Innovating Quality Education in Colleges and Improving the Professional Development of Young Teachers in Colleges

### 4.1. Innovative Quality Education in Colleges

#### 4.1.1. Integrate the Characteristics of Running a School and Clarify the Training Objectives of Quality Education

First of all, according to the regional characteristics of education, the school running characteristics of colleges and universities and the division of subject attributes, the quality education objective management system is established, the characteristics of education are further defined, and the quality education standards are proposed to strive to achieve the goal of the comprehensive development of information technology. Secondly, based on the needs of college students to grow and become talented, carefully designing the content of it is in line with the core socialist values and the development requirements of socialism with Chinese characteristics, establishing a spirit and benevolence and integrity as the main content. The traditional virtues and the noble character with the core of righteousness and morality as the focus of quality education, improve quality teaching.

RETRACTED

#### 4.1.2. Strengthen Top-Level Design and Improve the Quality Education Development Platform

School education should follow the basic law of the development and success of students of the National People's Congress, follow the logical order of from shallow to deep, from outside to inside, do a good job in the overall planning of school education, and implement comprehensive quality education in the whole process of quality education. First, the leading organs of higher education must pay attention to the education of undergraduates conceptually, fully guarantee the normal development of quality education at the levels of personnel, institutions, funds and measures, and establish a special quality education implementation guarantee plan to strengthen the strategic main role of quality education. Second, make use of network resources to establish channels for the development and improvement of quality education, and infiltrate educational ideas, means and skills into students' ideological mastery, knowledge mastery, vocational skills training, ideological and moral level, cultural quality, physical quality, and innovation ability. Third, based on the students' personal interests and hobbies, give full play to the main functions of campus practical teaching platforms such as professional knowledge practical quality education, excellent college students association practice activities, science and technology entrepreneurship experiments, and effective ways to further carry out quality education by using the practical teaching platforms inside and outside the school.

### 4.2. Improve the Career Development of Young Teachers in Colleges

#### 4.2.1. Improve the Teacher Promotion Evaluation System

The evaluation institutions for college teachers set up by colleges and universities are mainly established in accordance with the relevant provisions of the State Council and regions, and according to the work tasks and missions of colleges and universities. Therefore, for the evaluation institutions of university teachers, policy guidance is very important. The relevant education administrative departments of the state should, according to the current situation in the evaluation of college teachers and the current development direction and trend of the overall higher education, issue specific standards for the evaluation of college teachers. At present, the relevant regulations formulated by the government departments are relatively general, reflecting the principles of education management, but there is no specific operability. Listen to the suggestions of the front-line teachers, conduct repeated discussions, and put forward the detailed rules of the scoring method for reference.  Figure 5 shows the impact mechanism on their career development of them in colleges.

RETRACTED

#### 4.2.2. Pay Attention to the Training of Young Teachers

The school has been a focus on talent training. Based on the information of the actual investigation, the efforts and costs of introducing talents in colleges are relatively high, and the supporting young teacher training system has certain deficiencies. This situation is common in all colleges and universities. While paying attention to the introduction of talents, schools should not neglect the training of existing young teachers in schools. Schools must formulate supporting policies to realize systematic training modes and channels for young teachers.

Improve the supporting pre-job training mechanism, on the one hand, let teachers understand the school's organizational goals, organizational culture, and development direction, so that teachers can meet the school's development needs based on combining their advantages; on the other hand, young teachers should also be given more attention. With more training content and more intensive training requirements, teachers constantly guide teachers to strictly demand themselves and improve their professional ability and work literacy.

#### 4.2.3. Establish a Good Development Platform for Young Teachers

It is suggested that colleges and universities provide better training opportunities for young teachers and allocate senior teachers with rich teaching experience to the young teachers. By adopting face-to-face online courses, young teachers can quickly grasp and adapt to the new teacher's job, and promote the professional knowledge and management level of young teachers through sharing and exchanging teaching experience, thus realizing benign interactive teaching. Such an opportunity for young teachers to grow can be taught to them, and they can freely choose training programs according to the different needs of each teacher. This will also help each teacher to concentrate on developing their own advantages and achieving their own goals, and then improve their career development route.

RETRACTED

## 5. Conclusion

College teachers are an integral part of college talent resources. Excellent organizations are inseparable from the construction of talents, and the same is true for colleges and universities. The teaching staff has a significant impact on the future development of colleges and universities, and serves as a key force to enhance the vitality of running schools, enhance the potential of disciplines, strengthen innovation capabilities, and develop a new generation of outstanding talents. The cultivation of talents must have a certain environment, and similarly, the development of talents must also be supported by a corresponding environment. Colleges and universities, should comprehensively implement policies and take a multi-pronged approach, combine the conditions and characteristics of the school, and work together in terms of teachers and to cultivate compound talents who have both individual characteristics and meet it; cultivate students' learning awareness, promote the healthy development of student's physical and mental health, and reflect the meaning and value of quality education.

## Figures and Tables

**Figure 1:** Development of young teachers in colleges.

**Figure 2:** Market size and growth rate of China's quality education industry from 2017 to 2023.

**Figure 3:** The status quo of developing students' quality education in colleges at all levels.

**Figure 4:** The number of NS papers published by young teachers in colleges from 2003 to 2017.

**Figure 5:** Influence mechanism of career development of young teachers in colleges.

**Table 1:** The nine stages of Shien's career development theory.

Stage	Role	Main tasks and content
0–21: Growth, fantasy	Student	Identify your own needs, interests, abilities, and lay a solid foundation
16–25: The world of work	Applicants	Get involved and enter your career
16–25: Basic training	Intern	Understand and be familiar with the organization and recognize the organizational culture
17–30: Early career	Full member	Take responsibility for a successful first job assignment
25+: Mid-career	Full member, life member	Enter the management department through your own professional
35–45: Mid-career crisis	Supervisor, manager	Realistically assess your own progress
40 to retirement: Late careers	Key members, managers	Develop as a job coach
40 to retirement: Recession and departures	Different people decline or quit at different ages	Recognize reduced power, responsibility and status
Leave the organization or retire	Lose job	Form a certain sense of identity and adapt to changes in roles and life patterns

RETRACTED

**Table 2:** Liao Quanwen's “Three Three Three” Theory.

Stage		Individual work status	Occupational environment status
Output stage	Adaptation stage	Obey the arrangement of the leader, cooperate with colleagues, and perform well personally	Adapt to the working software and hardware environment
	Innovation stage	Take on tasks independently	Receive leadership and public recognition
	Re-adaptation stage	Get promoted for good work	Individuals adjust their mentality and adapt to the environment again

**Table 3:** H University full-time teachers' age-professional job statistics table.

generation	Positive height	Deputy Senior	Intermediate	Primary	Undetermined	Total
Under 25	0	0	0	2	0	2
26–30 years old	1	2	54	31	10	98
26–30 years old	16	60	108	4	2	190
26–30 years old	20	141	95	0	2	258
26–30 years old	45	157	67	2	2	273
26–30 years old	62	87	27	1	180	357
26–30 years old	93	98	28	0	1	220
26–30 years old	37	40	3		2	82
Over 60 years old	15	1	0	4	0	20
Total	289	586	382	44	199	1500

**Table 4:** Statistical table of feelings about the profession of teachers in colleges.

Frequency		Response		% of cases
		*N*	Percentage (%)	
Feelings about the teaching profession in colleges	Relatively easy	9	4.5	13.5
	Relatively busy	49	24.5	64.0
	Very stressed	35	17.5	45.5
	Have a sense of pride	38	19.0	49.5
	A sense of accomplishment	35	17.5	45.5
	Very motivated	29	14.5	37.5
	Relatively tired	4	2.0	4.5
	Other	1	0.5	1.0

Total	200	100		

**Table 5:** The factors that affect one's career development in order of importance.

Factors that affect your career development	Importance
Research level	4.85
Academic development	4.36
Teaching level	4.03
Interpersonal communication	3.46
Working environment	2.52
Other	0.1

## Data Availability

The labeled data set used to support the findings of this study is available from the corresponding author upon request.
